RETRACTED

# PBTNet: A New Computer-Aided Diagnosis System for Detecting Primary Brain Tumors

**DOI:** 10.3389/fcell.2021.765654

**Published:** 2021-10-15

**Authors:** Si-Yuan Lu, Suresh Chandra Satapathy, Shui-Hua Wang, Yu-Dong Zhang

**Affiliations:** ^1^School of Computing and Mathematical Sciences, University of Leicester, Leicester, United Kingdom; ^2^School of Computer Engineering, KIIT Deemed to University, Bhubaneswar, India

**Keywords:** computer-aided diagnosis, magnetic resonance imaging, primary brain tumors, brain cells, convolutional neural network, extreme learning machine

## Abstract

Brain tumors are among the leading human killers. There are over 120 different types of brain tumors, but they mainly fall into two groups: primary brain tumors and metastatic brain tumors. Primary brain tumors develop from normal brain cells. Early and accurate detection of primary brain tumors is vital for the treatment of this disease. Magnetic resonance imaging is the most common method to diagnose brain diseases, but the manual interpretation of the images suffers from high inter-observer variance. In this paper, we presented a new computer-aided diagnosis system named PBTNet for detecting primary brain tumors in magnetic resonance images. A pre-trained ResNet-18 was selected as the backbone model in our PBTNet, but it was fine-tuned only for feature extraction. Then, three randomized neural networks, Schmidt neural network, random vector functional-link, and extreme learning machine served as the classifiers in the PBTNet, which were trained with the features and their labels. The final predictions of the PBTNet were generated by the ensemble of the outputs from the three classifiers. 5-fold cross-validation was employed to evaluate the classification performance of the PBTNet, and experimental results demonstrated that the proposed PBTNet was an effective tool for the diagnosis of primary brain tumors.

## Introduction

The brain is the most sophisticated organ in the human body, so brain tumor, the uncontrolled growth of brain cells, is one of the deadliest diseases. People of any age can be affected by brain tumors. Unfortunately, the causes of most brain tumors are still unknown. The risk factors related to brain tumors include age, radiation, and genetic condition. So far, there are over 120 different brain tumors documented. However, they can be classified into two groups: primary brain tumors and metastatic brain tumors. Primary brain tumors develop from brain cells in normal brains. The types of primary brain tumors are dependent on the cells of origin. For instance, the primary brain tumors developed from glial cells are called gliomas. Also, some tumors originate from multiple types of cells, such as oligo-astrocytoma. The exact causes of primary brain tumors are still under research, but some factors are believed to be related to the tumors, including age, radiation, and genetic conditions.

RETRACTED

The growth of tumors is uncontrollable, accurate diagnosis of primary brain tumors is significant and beneficial for the treatment, especially at their early stage. Because the earlier the patient receives medical treatment, the higher is the chance of his/her survival. Currently, most diagnosis results are made by medical imaging. For primary brain tumor detection, magnetic resonance (MR) imaging is the first choice because it can provide better imaging results for soft tissues than computed tomography (CT). However, manual interpretation of MR images (MRIs) poses a heavy burden for the specialists, and it is unavoidable to suffer from high inter- and intra-observer variance. Computer-aided diagnosis (CAD) received more and more attention from both academia and industry because CAD systems can assist the specialists in their clinical diagnosis. With the unprecedented development of computer vision technology and artificial intelligence, CAD systems can implement automatic analysis of brain MRIs and output the diagnosis results, which can be verification of the manual analysis. Over the recent decade, an ocean of CAD methods has been proposed for the diagnosis of brain tumors.

Arunkumar et al. (2018) proposed a CAD system to detect brain tumors which can be used for both segmentation and classification of brain MRIs. Fourier transform was employed to enhance the quality of brain MRIs. Then, they utilized pixel-level features for segmentation. Finally, geometry and texture features including histogram of oriented gradients (HOG) were extracted for identification. Amin et al. (2019a) first pre-processed the MRI slices using a set of high pass and median filters to obtain smoother images with highlighted edges. Then, a seed-growing algorithm was proposed to segment the images, and a stacked sparse autoencoder was trained to classify the images as tumor or healthy. Extensive experiments were carried out and the results demonstrated that their method achieved promising classification ability. Later, Amin et al. (2019b) suggested using the long short-term memory (LSTM) model and Gaussian filters for the classification of brain tumors in MRIs. Chatterjee and Das (2019) put forward a hybrid method to classify gliomas as benign or malignant. Several filters were used for pre-processing, and the segmentation was implemented using clustering algorithms. Combined features including gray-level co-occurrence matrix and laws energy texture features were extracted to form the feature vector. Finally, type-II fuzzy logic and adaptive neuro-fuzzy inference were ensembled for classification. The proposed system was evaluated on public datasets and yielded satisfactory results. Aboelenein et al. (2020) proposed an improved U-Net with two tracks for brain tumor segmentation. The final segmentation results were obtained by merging the two tracks. Focal loss and generalized dice were also employed to handle the class-imbalanced problem. Hirata et al. (2020) explored the factors related to the time for the diagnosis of pediatric brain tumor and discovered that it required a longer time to accurately diagnose when the pediatric brain tumor patients were with visual disturbance or endocrine disorder. Hollon et al. (2020) put forward a near real-time intra-operation brain tumor diagnosis system based on stimulated Raman histology images. They used over 2.5 million images to train their CNN model. The testing results revealed that their CNN model can achieve good brain tumor diagnosis performance which was comparable to pathologist-based analysis. Additionally, they put forward a segmentation algorithm for the stimulated Raman histology images to get tumor regions. Hu and Razmjooy (2020) removed the noise from brain MRIs and implemented segmentation using Kapur thresholding and mathematical morphology. Afterward, a set of image features were extracted including entropy, energy, eccentricity, correlation, etc, and a deep belief network (DBN) was trained for classification. An improved seagull optimization algorithm was proposed to train the DBN and find the best subset of features simultaneously. Huang et al. (2020) presented a CAD system to classify pathological brains from normal ones in MRIs. Initially, a rectification algorithm was proposed the adjust the axis of the images automatically. Then, they put forward a deep convolutional neural network (CNN) model with differential feature map blocks and squeeze-and-excitation blocks for classification. Experiment results suggested that the differential feature block can be beneficial to improve classification performance. Kalaiselvi et al. (2020) proposed a brain tumor diagnosis system composed of three phases. In phase I, the brain MRIs were divided into 8 × 8 blocks, and statistical features were extracted from the blocks. Then, an infinite feature selection algorithm was employed to obtain the optimal feature set, and a support vector machine (SVM) was trained to classify them as tumor or non-tumor. In phase II, segmentation of the MRIs was implemented using a length region growing algorithm. The final phase III aimed for post-processing and estimation. The classification accuracy of their system was 97%. Kaplan et al. (2020) suggested using two modified local binary patterns to generate features from brain MRIs. Then, they trained several classifiers for classification including *k*-nearest neighbors, artificial neural network, random forest, etc. The best accuracy was 95.56%. Khalil et al. (2020) proposed to extract the tumor edges from 3D MRIs with a dragonfly algorithm. Then, they employed a level set segmentation algorithm to get the tumor regions based on the edges. Khan et al. (2020) proposed their brain tumor detection method based on the Internet of medical things. They extracted a set of statistical features from brain MRIs, i.e., perimeter, cell count, angle, area, density, solidity, and size. A partial tree algorithm was proposed for recognition, which was compared with random forest, random tree, and naïve Bayesian classifier in their experiments. Natekar et al. (2020) found that the interpretability of current brain tumor segmentation models was weak although they could produce promising segmentation results. Hence, they attempted to provide a visualized explanation that is understandable for human. Noreen et al. (2020) proposed to employ two pre-trained CNN models: Inception-v3 and DenseNet-201 for brain tumor classification from MRIs. They utilized the two deep models for representation generation. The features were obtained from the intermediate layers of the two models and were concatenated, respectively. A softmax layer served as the classifier. Purushottam Gumaste and Bairagi (2020) leveraged statistical features and an SVM for brain tumor segmentation in MRIs. Saba et al. (2020) first segment the brain MRIs using the Grab cut algorithm. Then, they employed a VGG for feature extraction, and the features from VGG were concatenated with shape and texture features. A maximum entropy feature selection algorithm was proposed to eliminate the redundant features. They trained multiple classifiers including k-nearest neighbors, decision tree, SVM, etc. Sharif et al. (2020) presented a triangular fuzzy median filtering for tumor segmentation. Similar texture features were computed and an extreme learning machine (ELM) was trained for the final prediction of the labels. Xu et al. (2020) employed median filtering for noise reduction, Kapur thresholding and morphological operations for segmentation, discrete wavelet transform and gray-level co-occurrence matrix for feature extraction, and a DBN for classification of the brain tumors. They also proposed an enhanced moth search algorithm to optimize the parameters in the DBN. Yin et al. (2020) improved the whale optimization algorithm with chaotic theory and logistic method. The improved whale optimization algorithm was used to train a multi-layer perceptron to identification brain tumors in MRIs. Lin et al. (2021) used U-Net as the backbone model and presented their aggregation and attention network for brain tumor segmentation. In their model, down-sampling and up-sampling layers were added to deal with information loss. Multi-scale and multi-receptive blocks were also embedded in their model. Their model achieved state-of-the-art segmentation performance. Ma and Zhang (2021) proposed a lightweight CNN model based on CSPDarknet for brain tumor detection, which achieved good balance between accuracy and efficiency. Their model produced an accuracy of 97% and can be deployed on mobile devices. Sadad et al. (2021) implemented brain tumor segmentation based on U-Net and ResNet-50. They proposed to use transfer learning with pre-trained CNN models for brain tumor classification. Zhang et al. (2021) proposed a multi-encoder net with a novel loss function for brain tumor segmentation in 3D MRIs. The drawbacks of these state-of-the-art approaches are summarized in Table 1.

RETRACTED

**TABLE 1:** Drawbacks of state-of-the-art approaches.

**Method**	**Drawbacks**
Arunkumar et al., 2018	The sensitivity was low for brain tumor detection, which was only 89%.
Amin et al., 2019a	The classifier was a softmax layer, which was too simple.
Amin et al., 2019b	The dataset was too small to train their deep model for classification.
Chatterjee and Das, 2019	Handcrafted image features may suffer from low transferability.
Aboelenein et al., 2020	The performance of their method was just slightly better than U-Net.
Hirata et al., 2020	Their conclusion from the small dataset may not be general.
Hollon et al., 2020	The training of their CNN was tedious.
Hu and Razmjooy, 2020	The swarm intelligent optimization required too much memory to train deep models.
Huang et al., 2020	The improvement was only less than 2% compared with the baseline model.
Kalaiselvi et al., 2020	The classification performance was dependent on the patch size.
Kaplan et al., 2020	Handcrafted image features may suffer from low transferability.
Khalil et al., 2020	The swarm intelligent optimization required too much memory.
Khan et al., 2020	Handcrafted image features may suffer from low transferability.
Natekar et al., 2020	Their conclusion was only based on limited experiments.
Noreen et al., 2020	The improvement was too small compared with the baseline model.
Purushottam Gumaste and Bairagi, 2020	Handcrafted image features may suffer from low transferability.
Saba et al., 2020	The classifier can be further optimized.
Sharif et al., 2020	Handcrafted image features may suffer from low transferability.
Xu et al., 2020	They didn’t compare their method with other state-of-the-art methods.
Yin et al., 2020	The swarm intelligent optimization required too much memory.
Lin et al., 2021	The improvement was too small compared with the baseline model.
Ma and Zhang, 2021	The accuracy of their model was only marginally better than the baseline method.
Sadad et al., 2021	Their dataset was class-imbalanced.
Zhang et al., 2021	Their method was obviously worse than one previously published method.

From the above analysis, it can be discovered that these CAD systems can produce accurate brain tumor classification results, but their performance is not ideal. Most of these state-of-the-art systems either used traditional machine learning classifiers with handcrafted features or employed deep CNN models for classification and recognition. However, handcrafted features, such as statistical features and texture features, are less transferrable. On the other side, deep CNN models contain massive parameters, and it may cause overfitting to train CNN models on medical image datasets, which are usually composed of only a small number of images. To cope with these problems, we present a new model for the classification of primary brain tumors called PBTNet. We select the pre-trained ResNet-18 as the backbone model in the PBTNet, and the backbone model serves as the feature extractor which is fine-tuned on the brain MRI dataset. The classifier in the proposed PBTNet is an ensemble of three randomized neural networks (RNNs): Schmidt neural network (SNN), random vector functional-link (RVFL), and extreme learning machine (ELM), which are all classical single hidden layer feedforward neural networks. The number of parameters in the RNNs is intensely smaller than that of a deep CNN model. Therefore, the overfitting problem can be avoided. Extensive experiments are conducted for performance evaluation of the PBTNet, and the results suggested that our PBTNet can produce accurate predictions of brain MRIs.

RETRACTED

The remainder of this study is organized as follows. Section “Materials and methods” is about the materials in the experiments. The presentation of our PBTNet is given in Section “Methodology.” The settings in the experiments are demonstrated in Section “Experiment design.” The experimental results and analysis are provided in Section “Results and discussion.” Section “Conclusion” concludes this paper.

## Materials and Materials

We obtained our brain MRIs for evaluation experiments from a public dataset available on the Kaggle website.^1^ We only included the slices of the brain MRIs in the transaxial view and consequently collected 276 slices of primary brain tumor (glioma) and 325 non-tumor samples in our dataset. The resolution of these images varied from 200 × 200 to 600 × 600. Some slices in our dataset were presented in Figure 1, where the left four images were primary brain tumors and the right four ones were non-tumor.

**FIGURE 1:** MRI slices in our dataset **(A)** Primary brain tumor samples. **(B)** Non-tumor samples.

## Methodology

Computer-aided diagnosis systems are usually based on computer vision technology and machine learning. For image classification, feature extraction is a necessary and important procedure because images contain excessive information which can increase the computational complexity dramatically. Handcrafted features were often used decades ago, such as statistical features and texture features. However, as deep learning models become the predominant method in artificial intelligence, CNN models have been successfully applied in computer vision tasks. Because the convolution and pooling layers in the CNNs can implement high-level representation learning automatically after training. The convolution filters serve as local perspectives, which substantially reduces the volume of parameters in the models. Meanwhile, the pooling operations can further reduce the dimension of the feature maps while maintaining predominant information. Therefore, more and more researchers and practitioners have poured their efforts to propel the performance of CNN models, and a sea of CNN models have been proposed, such as AlexNet (Krizhevsky et al., 2012), VGG (Simonyan and Zisserman, 2015), ResNet (He et al., 2016), DenseNet (Huang et al., 2016), MobileNet (Sandler et al., 2018), SqueezeNet (Iandola et al., 2016), EfficientNet (Tan and Le, 2019), etc. Hence, we attempt to utilize CNN models to detect primary brain tumors in MRIs. The workflow of the proposed PBTNet is presented in Figure 2. Initially, a ResNet-18 pre-trained on the ImageNet dataset is selected as the backbone model of the PBTNet. Then, the pre-trained ResNet-18 is modified and fine-tuned on the brain MRIs, and the last 4 layers are replaced by three RNNs: SNN, RVFL, and ELM. So, the ResNet-18 can be regarded as the feature extractor in the PBTNet. Afterward, the three RNNs are trained with features from the backbone model. Finally, the output of the PBTNet is obtained using the majority voting-based ensemble of the outputs from the three RNNs. The PBTNet is evaluated by 5-fold cross-validation (CV) to get the average classification performance for fair comparison. The detailed presentation of the PBTNet is given in the rest of this Section.

**FIGURE 2:** Flowchart of our PBTNet.

RETRACTED

### Transferred ResNet for Feature Extraction

There are several milestones in the development history of CNN models in the recent decade. First of all, the success of AlexNet (Krizhevsky et al., 2012) is the curtain-raiser of the prosperity in deep learning research. Then, the advent of ResNet (He et al., 2016) can be regarded as the second milestone because the shortcut connections in the residual blocks make it easier to train deeper CNN models effectively. After that, the residual mechanism can be found in almost every CNN model. The idea of shortcuts is simple, but the mathematical principles are profound.

In a vanilla CNN without shortcuts, the training of the model is to tune the parameters to make the mappings from the input layer to the output layer more and more accurately. As the activation functions in CNN models are usually the rectified linear unit (ReLU):


(1) ReLU⁢(x)=max⁢(0,x)

which is non-linear, researchers discovered that the non-linear layers have difficulty in implementing identity mapping during the training iterations. As a result, it is hard to train CNN models, especially when the CNNs get deeper layers. To handle this problem, the residual mechanism is proposed. An example of a residual block is shown in Figure 3. The original target mapping function of these convolutional layers is denoted as *f*(*x*). With the shortcut, these layers can be trained to approximate the residual function:


(2) res⁢(x)=f⁢(x)-x

Consequently, we can obtain the converted target function as:


(3) f⁢(x)=res⁢(x)+x

As a result, the training of these layers becomes more effective when approximating identity mappings because the activations can be shrunk to zero with the shortcut.

**FIGURE 3:** A shortcut in a CNN.

Therefore, we propose to use the ResNet-18 as the backbone model in the PBTNet. We believe that transfer learning is a better choice to use deep models than training from scratch for a specific image classification task. Because the CNN models pre-trained on the ImageNet dataset have acquired the ability to generate high-level image representations in the latent space which can be transferred to other image classification problems. Nevertheless, some modifications should be made on the ResNet-18 in respect to the difference between the ImageNet dataset and the brain MRI dataset, as is demonstrated in Figure 4. The original “FC 1000” is replaced by the “FC 2” as there are only two categories of images in our brain MRI dataset. Further, an “FC 25” is inserted into the model to mitigate the difference of dimensions between the “Pool 5” and “FC 2.” The modified ResNet-18 is fine-tuned on our brain MRI dataset, and the last four layers are replaced by three RNNs to achieve better classification performance. Therefore, the ResNet-18 only serves as the feature extractor in the proposed PBTNet, and the “FC 256” is the feature layer.

RETRACTED

**FIGURE 4:** Transfer learning using ResNet-18 (“FC”: fully connected).

### Ensembled Randomized Neural Networks for Classification

Convolutional neural network (CNN) models work well on big datasets, such as the ImageNet dataset. However, for small datasets, overfitting is likely to happen. Therefore, we propose to replace the last four layers in the ResNet-18 with three randomized neural networks for classification: Schmidt neural network (SNN) (Schmidt et al., 1992), random vector functional-link (RVFL) (Pao et al., 1994), and extreme learning machine (ELM) (Guang-Bin et al., 2006). The parameters in the layers of ResNet-18 are frozen when training the RNNs, so the ResNet-18 can be regarded as the image representation generator in our PBTNet. The structures of the three RNNs are presented in Figure 5. It can be found that the SNN and ELM are similar, and the only difference is that the SNN has biases in the output layer while the ELM doesn’t have output biases. The RVFL differs from the other two RNNs obviously in that it has shortcut connections directly from the input layer to the output layer.

**FIGURE 5:** Structures of three RNNs **(A)** SNN, **(B)** RVFL, **(C)** ELM.

Although the structures of the three RNNs are different, the training of the three RNNs has a unified form, which all can be summarized in three steps. Given a training dataset with its *i*-th sample as (***x*_*i*_**,***y*_*i*_**),


(4) xi=(xi1,…,xin)T∈ℝn,i=1,…,N

(5) yi=(yi1,yi2,…,yim)T∈ℝm,i=1,…,N

The training algorithm of the three RNNs is presented as follows. First, the weights and biases from the input layer to the output layer are assigned with random values, and they don’t change during the training. Then, the output matrix of the hidden layer with $\hat{N}$ nodes can be computed using the training set:

For SNN:


(6) $${\text{H}}_{S\,N\,N}=\sum_{j=1}^{\hat{N}}g\,\left(\alpha_{j}\,{\text{x}}_{i}+\beta_{j}\right),i=1,\ldots ,N$$

For RVFL, the situation is a bit different, the matrix is a concatenation of the input feature set and the random hidden mappings as:


(7) $${\text{H}}_{\mathrm{RVFL}}=\mathrm{concat}\,\left(X,R\right)$$

where **X** = (***x*_1_**,, ***x*_*N*_**)^T^ represents the input matrix and the R is:


(8) $$\text{R}=\sum_{j=1}^{\hat{N}}g\,\left(\alpha_{j}\,{\text{x}}_{i}+\beta_{j}\right),i=1,\ldots ,N$$

For ELM:


(9) $${\text{H}}_{\mathrm{ELM}}=\sum_{j=1}^{\hat{N}}g\,\left(\alpha_{j}\,{\text{x}}_{i}+\beta_{j}\right),i=1,\ldots ,N$$

Finally, the output weights can be obtained using pseudo-inverse:


(10) $$\lambda ={\text{H}}_{\mathrm{NET}}^{†}\,\text{Y},\mathrm{NET}=\mathrm{RVFL},\mathrm{or}\,\mathrm{ELM}$$

where ${\text{H}}_{\mathrm{NET}}^{†}$ denotes the pseudo-inverse matrix of **H_NET_** and **Y** = (***y*_1_**, …, ***y*_*N*_**)^T^ is the ground-truth label matrix of the training set. For SNN with output biases, the equation becomes:


(11) $$\left(\lambda ,\gamma \right)={\text{H}}_{\mathrm{SNN}}^{†}\,\text{Y}$$

where ${\text{H}}_{\mathrm{SNN}}^{†}$ is the pseudo-inverse matrix of (HSNN1).

RETRACTED

In this way, the training of three RNNs in the PBTNet finishes within merely three steps, which is fast. To further improve the robustness of the system, we employ the majority voting-based ensemble of the three RNNs. As the primary brain tumor detection is a binary classification problem, there is always a majority label in the predictions of the three RNNs for each brain MRI.

## Experiment Design

The proposed PBTNet is developed based on MATLAB 2021a with the deep learning toolbox. The evaluation results are all obtained using 5-fold cross-validation on a laptop with i7 CPU and GTX1060 GPU.

### Evaluation Metrics

To evaluate the classification performance of the proposed PBTNet, five metrics are employed: accuracy (ACC), sensitivity (SEN), specificity (SPE), precision (PRE), and F1-score (F), which can be computed by


(12) $$\text{ACC}=\frac{\mathrm{TP}+\mathrm{TN}}{\mathrm{TP}+\mathrm{TN}+\mathrm{FP}+\mathrm{FN}}$$

(13) $$\text{SEN}=\frac{\text{TP}}{\mathrm{TP}+\mathrm{FN}}$$

(14) $$\text{SPE}=\frac{\text{TN}}{\mathrm{TN}+\mathrm{FP}}$$

(15) $$\mathrm{PRE}=\frac{\text{TP}}{\mathrm{TP}+\mathrm{FP}}$$

(16) $$\text{F}=2\times \frac{\mathrm{PRE}\times \mathrm{SEN}}{\mathrm{PRE}+\mathrm{SEN}}$$

In which the TP, TN, FP, and FN denote true positive, true negative, false positive, and false negative, respectively.

### Hyper-Parameter Settings

The hyper-parameter settings in our PBTNet are demonstrated in Table 2. For fine-tuning the backbone model, the mini-batch size is only 10 because our brain MRI dataset is small with only hundreds of samples of two categories. The max-epoch is set as 2 to avoid overfitting. The learning rate is 1e-4, which is a conventional setting. The only pre-defined hyper-parameter in the three RNNs is the number of hidden nodes, $\hat{N}$, which is set as 400 because the input dimension of the RNNs is 256. The random mapping from lower dimension to higher dimension space is beneficial for the classification.

**TABLE 2:** Hyper-parameter settings in the PBTNet.

**Hyper-parameter**	**Value**
Mini-batch size	10
Max-epoch	2
Initial learning rate	1e-4
$\hat{N}$	400

RETRACTED

## Results and Discussion

### The Performance of the PBTNet

The classification performance of the proposed PBTNet based on 5-fold cross-validation is presented in Table 3. The total running time of the 5-fold cross-validation is 383.12 s. It can be revealed that the PBTNet achieved a sensitivity of 99.64%, which was outstanding because sensitivity can be regarded as the most important metric for clinical diagnosis. Meanwhile, the accuracy and F1-score were both above 96%. Together, the PBTNet is an effective tool to detect primary brain tumors in MRIs.

**TABLE 3:** Performance of the PBTNet based on 5-fold cross-validation (unit: %).

	**ACC**	**SEN**	**SPE**	**PRE**	**F**
Fold 1	97.52	100.00	95.59	94.64	97.25
Fold 2	97.50	100.00	95.59	94.55	97.20
Fold 3	96.67	100.00	94.20	92.73	96.23
Fold 4	98.33	98.18	98.46	98.18	98.18
Fold 5	95.00	100.00	91.55	89.09	94.23
Average	97.00	99.64	95.08	93.84	96.62

### Effects of Different Backbone Models in the PBTNet

We tested the performance of our PBTNet with other famous pre-trained CNNs as backbones. The results based on 5-fold cross-validation were given in Table 4 and Figure 6. The classification performance of the PBTNet with different backbones was close except the one based on AlexNet. The PBTNet with ResNet-18 as the backbone model produced the best sensitivity, F1-score, and overall accuracy. The shortcut connections in the ResNet-18 contributed to the convergence, and ResNet-18 was more lightweight than ResNet-50 so it was more suitable for our small dataset. Therefore, we utilized the ResNet-18 as the backbone of our PBTNet.

**TABLE 4:** Performance of the PBTNet with different backbones based on 5-fold cross-validation (unit: %).

**Backbone**	**ACC**	**SEN**	**SPE**	**PRE**	**F**
AlexNet	89.68	94.86	86.59	82.22	87.91
MobileNet v2	96.34	98.16	95.06	98.83	95.89
ResNet-18	97.00	99.64	95.08	93.84	96.62
ResNet-50	95.84	96.04	95.76	94.93	95.45
EfficientNet	94.84	98.05	92.52	90.57	94.15

**FIGURE 6:** Performance of the PBTNet with different backbones based on 5-fold cross-validation (unit: %).

### Transfer Learning Versus Training From Scratch

The initial weights of the backbone models were important for the final classification of our PBTNet. Hence, we experimented on the classification performance of the PBTNet with pre-trained ResNet-18 and untrained ResNet-18. The results based on 5-fold cross-validation were provided in Table 5. It is obvious that the PBTNet based on pre-trained ResNet-18 performed better than that with untrained ResNet-18. So, it can be inferred that the weights in the ResNet-18 obtained from the ImageNet dataset contributed to the higher diagnosis accuracy. Although the brain MRI dataset was obviously different from the ImageNet dataset, there can be similarities in the latent feature space. Therefore, transfer learning is a better option for the backbone model in the PBTNet than training from scratch.

RETRACTED

**TABLE 5:** performance of the PBTNet with pre-trained ResNet-18 and untrained ResNet-18 based on 5-fold cross-validation (unit: %).

**Backbone**	**ACC**	**SEN**	**SPE**	**PRE**	**F**
Untrained ResNet-18	92.68	95.39	90.86	88.40	91.67
Pre-trained ResNet-18	97.00	99.64	95.08	93.84	96.62

### Effects of Classifier Ensemble

We demonstrated the results of the three RNNs and compared them with the PBTNet which was the ensemble of the three models. The statistics are presented in Table 6 and Figure 7. The accuracy, sensitivity, and F1-score of the ensembled model, PBTNet, were all better than the three RNN based models. As for the specificity and precision, PBTNet also outperformed the ResNet-18-RVFL and ResNet-18-ELM. In conclusion, the ensemble mechanism based on majority voting can improve the classification performance of our model for primary brain tumor detection.

**TABLE 6:** Comparison of the proposed models based on 5-fold cross-validation (unit: %).

	**ACC**	**SEN**	**SPE**	**PRE**	**F**
ResNet-18-SNN	96.51	97.40	95.83	94.92	96.13
ResNet-18-RVFL	96.84	99.27	95.06	93.84	96.44
ResNet-18-ELM	95.84	98.10	94.15	92.75	95.34
PBTNet	97.00	99.64	95.08	93.84	96.62

**FIGURE 7:** Comparison of the four proposed models (unit: %).

### Explainability of the PBTNet

The explainability of deep neural networks is a significant facet of deep learning because deep models are more like black boxes in applications. We cannot figure out how they make predictions. Gradient-weighted class activation mapping (Grad-CAM) (Selvaraju et al., 2017) offered an approach to visualize the attention of the deep networks when they predicted. We presented two Grad-CAMs of the PBTNet on primary brain tumor MRIs in Figure 8. The red regions were where the attention of the PBTNet while the blue regions were believed to be less relative with the predictions by the model. It can be discovered that the tumors were within the red regions. Therefore, the proposed PBTNet was able to capture the tumors in brain MRIs.

**FIGURE 8:** Grad-CAMs of primary brain tumor MRIs.

### Comparison With Other State-of-the-Art Systems

We compared the proposed PBTNet with other state-of-the-art CAD systems for brain tumors and abnormalities including RBFNN (Lu et al., 2016), CNN (Sajjad et al., 2019), DCNN (Islam and Zhang, 2018), Feature ensemble (Saba et al., 2020), and Patches + SVM (Kalaiselvi et al., 2020). The results were given in Table 7 and Figure 9. Our PBTNet yielded the best accuracy, sensitivity, and F1-score in the listed methods. Meanwhile, for specificity and precision, it also ranked second, and the difference was very close to the highest values. The comparison suggested that our PBTNet is effective and accurate to detect primary brain tumors in MRIs. Deep CNN models can generate high-level image representations automatically, but overfitting may happen when they are applied on small datasets. The reasons for the good performance of the proposed PBTNet can be two-fold. First, the pre-trained ResNet-18 can generate beneficial features from the brain MRIs with only 2 epochs of training. Second, the RNNs are suitable for the classification of small datasets, and the ensemble based on majority voting further boosted the classification accuracy and improved the robustness of the PBTNet.

RETRACTED

**TABLE 7:** Comparison with state-of-the-art methods (unit: %).

**Methods**	**ACC**	**SEN**	**SPE**	**PRE**	**F**
RBFNN (Lu et al., 2016)	95.44	95.89	92.78	-	-
CNN (Sajjad et al., 2019)	94.58	88.41	96.12	-	-
DCNN (Islam and Zhang, 2018)	93	93	-	94	92
Feature ensemble (Saba et al., 2020)	91.74	95.08	87.33	-	-
Patches + SVM (Kalaiselvi et al., 2020)	83.90	98.46	-	-	-
PBTNet (ours)	97.00	99.64	95.08	93.84	96.62

**FIGURE 9:** Comparison with state-of-the-art methods (unit: %).

## Conclusion

In this study, We proposed a novel primary brain tumor diagnosis system based on brain MRIs. The proposed PBTNet employed the pre-trained ResNet-18 as the backbone model for feature extraction and used three RNNs: SNN, RVFL, and ELM for classification. The final predictions of the PBTNet were generated by the ensemble of the outputs from the three RNNs. 5-fold cross-validation was employed to evaluate the performance of the PBTNet and the average accuracy was 97.00%, which was better than five state-of-the-art methods.

In the future, we shall collect more samples to re-test the model. We will also try to develop cell-based classification CAD systems to implement more accurate diagnoses. In addition, the tumors can develop with time, so it can be beneficial for tumor diagnosis to analyze longitudinal data. Moreover, brain segmentation is also an important topic in clinical diagnosis, which can locate the lesions. Therefore, we shall pay more attention to brain segmentation in MRIs in the future.

## Data Availability Statement

The original contributions presented in the study are included in the article/supplementary material, further inquiries can be directed to the corresponding authors.

## Author Contributions

S-YL: conceptualization, methodology, software, data curation, writing – original draft, visualization, and funding acquisition. SS: methodology, formal analysis, writing – original draft, and project administration. S-HW: validation, formal analysis, investigation, writing – review and editing, supervision, and funding acquisition. Y-DZ: methodology, validation, investigation, resources, writing – original draft, writing – review and editing, supervision, project administration, and funding acquisition. All authors contributed to the article and approved the submitted version.

RETRACTED

## Conflict of Interest

The authors declare that the research was conducted in the absence of any commercial or financial relationships that could be construed as a potential conflict of interest.

## Publisher’s Note

All claims expressed in this article are solely those of the authors and do not necessarily represent those of their affiliated organizations, or those of the publisher, the editors and the reviewers. Any product that may be evaluated in this article, or claim that may be made by its manufacturer, is not guaranteed or endorsed by the publisher.

## Footnotes

1
www.kaggle.com/sartajbhuvaji/brain-tumor-classification-mri
